# Prenatal diagnosis of an aberrant ductus venosus draining into the coronary sinus using two- and three-dimensional echocardiography: a case report

**DOI:** 10.1186/s12884-021-03870-x

**Published:** 2021-05-20

**Authors:** Yu Wang, Ying Zhang, Meilian Wang

**Affiliations:** 1 Department of Ultrasound, Shengjing Hospital of China Medical University, Liaoning Shenyang, China; 2 Department of Microbiology and Parasitology, College of Basic Medical Sciences, China Medical University, Liaoning Shenyang, China

**Keywords:** Ductus venosus, Coronary sinus, 3D, Fetus

## Abstract

**Background:**

Ductus venosus (DV) abnormalities may be associated with intracardiac or extracardiac deformities, chromosomal anomalies, and/or congestive heart failure. Aberrant DV connecting with the coronary sinus (CS) is rare and the prenatal diagnosis presents challenges for most examiners.

**Case presentation:**

A 35-year-old pregnant woman, gravida 2, para 1, was referred to our center at 27 gestational weeks for a full evaluation of fetal cardiac anomalies. Transverse scans indicated normal cardiac anatomy except for a dilated CS; we then scanned sagittal planes to clarify the reasons for the CS dilatation. High-definition flow imaging (HDFI) together with radiant flow (R-flow) imaging was used to delineate the aberrant DV returning to the CS, enabling the diagnosis. Three-dimensional (3D) technology was also used to obtain color-rendered images showing the spatial relationships of the vessels involved, thus confirming the two-dimensional (2D) diagnosis. Chromosomal analysis revealed a normal karyotype. The neonate appeared healthy and the echocardiogram showed a normal cardiac anatomy except for a dilated CS with the DV closed and imperceptible.

**Conclusions:**

The aberrant course of the DV returning to the CS was clearly demonstrable by traditional 2D echocardiography using HDFI and the R-flow technique. We deem it helpful to trace the inflow of the dilated CS to make the differential diagnosis. The 3D modality might also provide additional spatial information on the associated vessels and thereby assist in prenatal diagnosis.

**Supplementary Information:**

The online version contains supplementary material available at 10.1186/s12884-021-03870-x.

## Background

The ductus venosus (DV) is a small vessel that bridges the intraabdominal umbilical vein (UV) and the inferior vena cava near the latter’s entrance to the right atrium [1]. Examination of the DV is now an integral component of the 11-13-week ultrasonographic scan in addition to nuchal translucency (NT) measurements [1, 2]. A negative a-wave on the waveform of the DV suggests a high association with fetal congenital heart disease (CHD), especially when it appears together with tricuspid regurgitation [3]. Aberrant connections of the UV may also be present in the case of the absence of DV (ADV), which is considered to be related to a high incidence of chromosomal abnormalities [1, 2]. The DV may exist under other conditions, but with an aberrant course and vascular associations. We herein report a rare case of aberrant connection of the DV to the coronary sinus (CS), using new color imaging techniques. The combination of high-definition flow imaging (HDFI) and radiant flow (R-flow) show the route of the aberrant vessel to a greater degree. We also used a three-dimensional (3D) technique to demonstrate the corresponding vessel positions in space, which will allow a better understanding of the anatomy.

## Case presentation

A 35-year-old woman, gravida 2, para 1, was referred to our center after the detection of a dilated CS at a second trimester ultrasonographic examination. First trimester findings were reported to be unremarkable, and NT was 1.6 mm. A thorough examination was then performed by an experienced fetal echocardiographer to assess any potential cardiac anomaly at 27 weeks of gestation. The four-chamber view revealed a normal heart with symmetrical chambers and normal atrioventricular associations except for the presence of CS dilatation (Fig. 1). In addition, the bilateral outflow tract views and the three-vessel tracheal view showed no evidence of abnormalities. During transverse scanning, the echocardiographer undertook an extensive examination to determine the normal drainage of the pulmonary veins and the non-existence of a persistent left superior vena cava (LSVC). A further evaluation to determine the reasons for the dilatation of the CS was carried out by scanning around the CS. When the sound beam was turned to section through the parasagittal plane of the fetus, a slim vessel was visualized draining into the CS; this was confirmed to be an aberrant DV as it originated from the UV (Fig. 2). Two additional movie files show this in more detail (See Additional files 1 & 2: Video). Other major veins-including the UV, hepatic and portal veins, and the inferior vena cava-showed a normal course and drainage.

**Fig. 1:** Sonograms showing the symmetrical four chambers (**a**) and the dilated coronary sinus (**b**). CS: coronary sinus; DAO: descending aorta; L: left; LA: left atrium; LV: left ventricle; R: right; RA: right atrium; RV: right ventricle; SP: spine

**Fig. 2:** Sonograms in parasagittal view showing the aberrant course of the ductus venosus. A small vessel is visualized draining into the coronary sinus (CS) near the insertion point of inferior vena cava to the right atrium (**a**). This vessel (indicated by a hand mark) turns to be the ductus venosus (DV) as it connects with the umbilical vein (UV). The arrows indicate the route of UV-DV connections that cannot be shown by color imaging as the blood flow is vertical to the sound beam (**b**). The origin and aberrant course of DV (indicted by arrows) could be better shown in another perspective (**c**) HV: hepatic vein; LA: left atrium; RA: right atrium


**Additional file 1: Video.** Sonograms showing the ductus venosus draining into the coronary sinus. A small vessel is visualized draining into the coronary sinus near the insertion point of inferior vena cava to the rightatrium.**Additional file 2: Video.** Parasagittal view of sonograms showing the origin and aberrant course of the ductus venosus. The DV originates from the umbilical vein and then courses upward to the coronary sinus, parallel to the inferior vena cava.

To clarify the diagnosis, 3D cardiac volumes were acquired with sagittal sweeps using HDFI over the upper abdominal and thoracic regions. The acquisition time was 12.5 s, and the sweep angle was set to 35°. The volumes were immediately reconstructed and displayed in a cine loop in multiplanar mode and then stored for later offline analysis using PC software (4D Viewer, version 14.0; GE Medical Systems, Zipf, Austria). Adjusting and rotating the images in the three orthogonal planes were used to facilitate a better reconstruction of the 3D image. A combination of smooth-surface and gradient-light algorithms and postprocessing adjustments was adopted to improve the quality of the 3D color-rendered image. The origin, course, and final drainage of the DV were clearly shown in the 3D image. The spatial relationships of the associated vessels were also demonstrated (Fig. 3).

**Fig. 3:** Three-dimensional color-rendered image showing the course and the connection of the ductus venosus in space. CS: coronary sinus; DV: ductus venosus; IVC: inferior vena cava; RA: right atrium; HV: hepatic vein; UV: umbilical vein

Based on the two-dimensional (2D) and 3D diagnosis of an aberrant DV communicating with the CS, amniocentesis for karyotype determination was requested for the patient; the results revealed a normal karyotype. Normal fetal growth was revealed by follow-up examination at 32 weeks of gestation, and the remainder of the pregnancy and delivery was uneventful. The weight at birth was 3242 g, and the neonate appeared healthy with Apgar scores of 10/10. Postnatal echocardiography performed on day 7 showed a normal cardiac anatomy except for a dilated CS, and the DV was closed and imperceptible. No further abnormality was noted, and cardiac systolic function appeared normal.

## Discussion and conclusions

As a channel between the intrahepatic UV and inferior vena cava, the DV functions in the distribution of umbilical venous return in two principal aspects. First, the oxygenated blood is directed to enter the right atrium through this shortcut and then preferentially steams through the foramen ovale, which ultimately benefits the cephalic and coronary circulations [1, 4]. In addition, the DV contains smooth muscle and connective tissue throughout its length, which serve as a constricting “sphincter” to protect the fetus from placental overcirculation [5]. It is a relatively straightforward deduction, then, that unrestricted umbilical venous return to the right atrium would occur with ADV. This may follow two different routes: the extrahepatic umbilical venous drainage bypassing the liver and the intrahepatic umbilical venous drainage without liver bypass. In the first case, the UV may directly drain to the right atrium, iliac vein, the inferior vena cava, or less commonly to the left atrium [6, 7]. Under the other condition, the UV drains into the portal sinus in its usual manner without engendering the DV [8–10].

Previous studies [4, 5, 10] indicated that ADV exhibited some association with congenital heart disease (CHD). Perles et al. [5] reported that 20 % of fetuses with ADV exhibited a structural heart disease when these authors reviewed the literature, while Berg et al. [4] indicated a much higher incidence rate of 47.8 % for CHDs in ADV fetuses. Extracardiac anomalies were also reported in ADV fetuses, the incidence of which varied from 4.3 to 35 % according to different case series [4, 5]. In addition, fetuses with ADV were frequently reported to possess complex malformation syndromes and chromosomal anomalies [7, 9–11]. Investigators have suggested a favorable prognosis for fetuses with isolated ADV and intrahepatic umbilical venous drainage [4]. In contradistinction, ADV fetuses with extrahepatic umbilical venous drainage showed an apparently worse prognosis due to a strong association with agenesis of the portal venous system [12, 13]. Previous studies also indicated that ADV fetuses with liver bypass manifested a significant association with high-output cardiac failure, cardiomegaly, and hydrops fetalis due to chronic volume overload of the central venous system [6, 7]. The aforementioned factors all indicate the importance of detecting fetal DV.

It is rare during routine obstetric examinations to observe a dilated CS where it receives blood from the UV. This type of CS dilatation is the consequence of fetal venous anomalies that can be categorized into three types: (1) the UV drains into the CS directly with ADV; (2) the UV communicates with the CS via the LSVC associated with ADV; and (3) the UV joins the CS through an aberrant DV. We performed a complete literature review and found only 15 such cases since the year 2002; these cases-together with the current case-are summarized in Table 1. It is noteworthy that six of the eight fetuses presented with differing degrees of cardiomegaly when the UV directly joined the CS. In contrast, none of the six fetuses showed an enlarged heart when the UV converged with the CS via a DV, which shows its function as a constricting “sphincter”. Half of the fetuses with a direct UV-CS junction expressed intracardiac and/or extracardiac malformations. For the two UV-LSVC-CS communicating fetuses, one showed a mild extracardiac anomaly. We were intrigued that no untoward consequences were observed for any of the six fetuses with a DV-CS junction. We readily understand the favorable prognosis for these patients, as the distribution of UV blood flow was unaffected and the vasculature of the portal system remained normal; in addition, no umbilicosystemic shunt was present. The aforementioned factors assure normal fetal hemodynamics and no risk of heart failure, either before or after birth [20]. We stress that chromosomal tests should be performed for fetuses with ADV or aberrant DV connections. Karyotype analysis is also used in the majority of the studies of fetuses with ADV [5, 10, 16], while copy number variation (CNV) should be examined as a complementary modality as it may show possible chromosomal microdeletions/microduplications.

**Table 1:** Review of fetuses with umbilical drainage to the coronary sinus directly or through a ductus venosus

References	Case	Referral indication	GA at diagnosis	Venosus connection	Additional US findings	Color technique	Chromosomal anomaly	Outcome
Volpe et al (Italy) [10]	1	Suspected CHD	26	UV/CS	Cardiomegaly, anorectal malformations	CDFI	Normal	Alive after surgery
Chi et al (USA) [14]	2	Suspected CHD	20	UV/CS	RA dilatation	CDFI	NA	NNA
Perles et al (Israel) [5]	3	Cardiomegaly	24	UV/CS	PLSVC, cardiomegaly, TR	CDFI	Normal	NNA
Achiron et al (Israel) [15]	4	Ascites	24	UV/CS	CAPVS, No IVC, RLCV, mitral atresia	CDFI	NA	TOP
Shen et al (Israel) [16]	5	NA	23	UV/CS	Ebstein anomaly	3D HDFI, 3D B-flow	Normal	Alive after surgery
	6	NA	26	UV/CS	LSUA	3D HDFI, 3D B-flow	Normal	NNA
	7	NA	25	UV/CS	Cardiomegaly, TR, ASD, PLSVC	3D HDFI, 3D B-flow	Normal	Hyperammonemia
Jowett et al (UK) [17]	8	Absent corpus callosum	25	UV/CS	PRUV, agenesis of the corpus callosum, diaphragmatic hernia	CDFI	NA	NNA
McBrien et al (Canada) [18]	9	Suspected CHD	24	UV/LSVC/CS	Absent nasal bone, diaphragmatic eventration	NA	NA	NNA
	10	Suspected CHD	21	UV/LSVC/CS	Renal pelviectasis	NA	NA	NNA
Qian et al (China) [19]	11	Suspected CS dilatation	24	UV/DV/CS	None	CDFI, 3D B-flow	NA	NNA
Ben et al (France) [20]	12	Suspected atrial abnormality	32	UV/DV/CS	None	CDFI	NA	NNA
	13-14	Suspected atrial abnormality	NA	DV/CS	None	HDFI	NA	NNA
	15	Suspected atrial CS dilatation	NA	DV/CS	None	HDFI	NA	NNA
Wang et al^a^ (China)	16	Suspected CS dilatation	23	DV/CS	None	HDFI, R-flow, 3D HDFI	Normal	NNA

Abbreviations: *3D* three-dimensional, *ASD* atrial septal defect, *CAPVS* congenital agenesis of the portal venous system, *CDFI* color Doppler flow imaging, *CHD* congenital heart disease, *CS* coronary sinus, *DV* ductus venosus, *GA* gestational age, *HDFI* high definition flow imaging, *IVC* inferior vena cava, *RLCV* rudimentary left cardinal vein, *LSUA* left single umbilical artery, *LSVC* left superior vena cava, *PLSVC* persistent left superior vena cava, *PRUV* persistent right umbilical vein, *NA* not applicable, *NNA* neonatal alive, *RA* right atrium, *R-flow* radiant flow, *TR* tricuspid regurgitation, *TOP* termination of pregnancy, *US* Ultrasonographic, *UV* umbilical vein

^a^the current case

It is important to identify the variant responsible so as to clarify the reasons for the dilatation of the CS. In fact, a dilated CS easily attracts the attention of most screening sonographers when scanning the four-chamber view. The dilatation of the CS always serves as an indirect sign of cardiac deformities or variants; thus, a thorough scan should be performed to determine the origin of the venous inflow to the CS. We recommend parasagittal scanning around the CS, which usually ensures a clear diagnosis. If the inflow vein extends cephalically, it becomes the left innominate vein; however, if the inflow vein turns to the rear of the atrium when the sound beam rotates from the sagittal to the transverse view, the vessel might be the common pulmonary vein in the case of an anomalous pulmonary venous connection. If a vessel runs cephalically, running parallel to the inferior vena cava and finally joining the CS, it might be the aberrant DV. Further scanning to trace the vessel’s origin from the UV would confirm the diagnosis. The possible situations presented above regarding the inflow veins are illustrated in Fig. 4 to show the differential diagnoses of CS dilatation.

**Fig. 4:** Schemes showing the strategy of making a differential diagnosis of dilated coronary sinus. This is an original illustration. Tracing the inflow vein of the CS in parasagittal views assists in clarifying the reasons for its dilatation. If the inflow vein extends cephalically, it turns to be the left innominate vein in the case of a LSVC (**a**). If the inflow vein turns to the rear of the atrium when the sound beam is rotated from the sagittal view to the transverse view, the vessel might be the CPV in the case of an anomalous pulmonary venous connection (**b**). If a vessel runs cephalically, running parallel to the inferior vena cava and ultimately joining the coronary sinus, it may be the aberrant ductus venosus (**c**). CPV: common pulmonary vein; CS: coronary sinus; DV: ductus venosus; HV: hepatic vein; LA: left atrium; LSVC: left superior vena cava; PA: pulmonary artery; RA: right atrium

Different color-imaging techniques show the fetal vasculature in a multitude of ways. As a special bidirectional Doppler technique, HDFI can better display vessel perfusion and blood flow continuity than traditional color Doppler [21]. R-flow imaging is a novel technique in which the index of erythrocyte density in a certain area is converted into a height index and then superimposed upon the initial coding of color maps. In the current study, we clearly demonstrated the trajectory of the associated vessels by simultaneously using HDFI and R-flow, which depicted the flow with a sense of depth and with sharper edges than is possible with color alone [22].

The 3D technology has played a decidedly important role in fetal cardiac imaging since its introduction in 2003. Cardiac volumes obtained from a single sweep contain a large amount of information that enables 3D reconstructions using proper data processing [23]. In addition, volume acquisition with B-flow/color/HDFI provides a 3D reconstruction of favorable vessels and allows a comprehensive evaluation of complex anatomic details: these show anatomic realism in 3D color, highlight spatial relationships of the great vessels, and emphasizie the 3D effect of structures of interest with enhanced depth perception [22]. Although the use of 3D B-flow has been demonstrated in a previous report from our center regarding evaluations of DV-CS conjunction and associated vessels [19], 3D images derived from B-flow volumes cannot show the direction of flow [22]. The current report is thus the first to show an aberrant DV adjoining the CS using 3D HDFI, with an apparently improved effect relative to previous 3D B-flow images.

It is important to note that volumes acquired from a sagittal sweep may obtain much more information than acquisitions starting in a transverse plane when assessing the central veins, great arteries, and their connections to the heart [22]. The volume then is displayed in three orthogonal planes immediately after completion of acquisition. The ensuing 3D reconstruction based on the coronal plane and a posteroanterior visualization of the fetus thus produces a superior display of the associated vasculature [24]. The 3D-reconstructed image might also provide additional spatial information, allowing for better consultations with obstetricians and parents.

In summary, we herein report a rare case of aberrant DV draining into the CS. We also proposed a strategy to render a differential diagnosis for dilated CS by tracing the inflow veins using a sagittal scan. The use of novel color-imaging techniques and 3D reconstruction should facilitate the visualization and understanding of the aberrant course of this variant. Given its ease of application, we expect broad usage of 3D technology in future clinical practice.

## Data Availability

The datasets supporting the conclusions of this article are included within the manuscript (and its additional files). The authors would like to share raw anonymized video data related to the current study, which could only be used for personal study. The demanders may contact the corresponding author.

## Abbreviations

3D: Three-dimensional
ADV: Absence of ductus venosus
CHD: Congenital heart disease
CNV: Copy number variations
CS: Coronary sinus
HDFI: High-definition flow imaging
LSVC: Left superior vena cava
DV: Ductus venosus
NT: Nuchaltranslucency
R-flow: Radiant flow
UV: Umbilical vein
